RETRACTED

# A Rare Reason for Pelvic Pain in Pregnancy: Infectious Sacroiliitis

**DOI:** 10.1155/2015/690429

**Published:** 2015-05-12

**Authors:** Yasemin Cekmez, Ahmet Göçmen, Oğuz Arslan, Fatih Şanlıkan, Simge Bağcı Türkmen

**Affiliations:** Department of Obstetrics and Gynecology, Ümraniye Medical and Research Hospital, 34000 İstanbul, Turkey

## Abstract

*Introduction*. Although the incidence of pregnancy-associated sacroiliitis is low, it is associated with significant morbidity and mortality. Timely diagnosis of the disease is confusing due to its nonspecific clinical features. *Case*. A 28-year-old woman at 34 weeks of gestation with severe pain in her right buttock radiating down the backside of the right thigh was admitted to our hospital. White blood cell (WBC) count and C-reactive protein (CRP) were elevated. The pelvic magnetic resonance imaging (MRI) scan revealed right sacroiliitis. *Conclusion*. Infectious sacroiliitis should be considered as a differential diagnosis even in low-risk women who present with debilitating pelvic pain in pregnancy and medical treatment should not be delayed.

## 1. Introduction

Pelvis and sacroiliac joints (SIJs) undergo considerable changes during pregnancy that have an impact on the dynamic stability of the pelvis [1]. While symmetrically increased SIJs laxity related to pregnancy and hormonal changes during pregnancy is not associated with pain, asymmetric laxity of the SIJs seems to be associated with moderate to severe pregnancy-related girdle pain (PGP) and correlates well with the severity scales and clinical test for SIJ dysfunction [2, 3]. Due to pregnancy-related pelvic girdle pain, the clinical presentation of sacroiliitis is sometimes camouflaged. We describe a case of a 28-year-old pregnant woman who presented at 34 weeks of gestation with severe pain in her right buttock radiating down the backside of her right thigh related to right SIJ infectious sacroiliitis.

## 2. Case

A 28-year-old (gravidity 4, parity 1) pregnant woman at 34 weeks of gestation was referred to our emergency unit because of severe pain in her right buttock radiating down the backside of the right thigh. She reported that the pain in her right buttock began 16 days before. The pain was worsened during daily activities and she became almost restricted to the bed. She had no low back pain history. Due to the intensity of the pain, she could not sit or stand by herself. Her bladder and bowel functions were normal. On her neurologic examination, feet extensor and flexor muscles strength were bilaterally normal but pelvic girdle muscle strength (consisting of bilateral iliopsoas, pectineus, and sartorius muscles strength) was reduced. Deep tendon reflexes of the legs were brisk without sensory loss. On the right side, posterior pelvic pain provocation (PPPP) and the active straight leg rise (ASLR) tests were positive [1, 4]. On the left side, it was very difficult for the patient to perform the same tests. The fetus was in transverse position, with good vital signs; the cardiotocogram was reactive, with good variability and without uterine contraction. Fetal biometric measurements were compatible with 34 weeks' gestation and amniotic fluid index was normal.

RETRACTED

The patient was admitted to the hospital. Laboratory findings were as follows: hemoglobin levels 11.3 g/dL, platelets 180 × 109/L, increased white blood cell (WBC) count of 14.16 K/uL, increased erythrocyte sedimentation rate (ESR) of 30 mm/h, and increased C-reactive protein (CRP) level of 14.1 mg/dL (normal range: 0.0–8.1 mg/L). Blood cultures taken for persistent fever were negative (36.8°C).* Brucella* agglutination test,* Listeria* agglutination test, and sputum culture for tuberculosis were negative. Doppler ultrasound examination of both legs was performed to exclude deep venous thrombosis. An echocardiogram did not find any evidence of endocarditis. Because of pregnancy, we did not use radiographs of lumbar spine and the pelvis. Magnetic resonance imaging (MRI) of the SIJs revealed joint space widening and effusion of the right SIJ indicating acute right-sided sacroiliitis (Figure 1). Depending on the clinical, laboratory, and radiological findings, the patient was diagnosed with right infectious sacroiliitis. The patient received broad-spectrum antibiotics such as ertapenem and daptomycin. Ultrasound guided aspiration was planned but could not be performed, because the patient could not be positioned concerning the enlarged uterus. Biophysical profile was performed to observe the fetal status twice a week. A rehabilitation procedure was initiated so that the patient might regain her strength and mobility. A cesarean section was performed under general anaesthesia at 38 weeks' gestation and a 2910 g female fetus was delivered. Medical treatment was continued throughout postpartum period. She received additional teicoplanin and oral ciprofloxacin therapy for 15 days. She was discharged 18 days after delivery with normal laboratory findings with daily physical exercise therapy. Control computed tomography images of the SIJs revealed normal appearance (Figure 2). Currently, except mild discomfort on her right buttock, she has normal body movements and mobility without a sequel or restriction.

## 3. Discussion

The function of the sacroiliac joint is to reduce pelvic stress caused by changes in weight due to body movement. Hormonal effects of pregnancy permit relaxation of the ligaments supporting the sacrum and the pelvic bones. It has been hypothesized that sacroiliitis in pregnancy is associated with microscopic areas of injury on the joint surfaces produced by the changes during pregnancy [5].

RETRACTED

Sacroiliac joint infection is considered uncommon and usually related to trauma, illicit drug addiction, or underlying diseases [5]. In our patient's case, there was an unremarkable past medical history and she denied a history of trauma or drug abuse. The presence of sacroiliitis without predisposing conditions and the nonspecific clinical presentation may delay diagnosis, especially when considering that lower back pain is a common symptom in pregnancy and postpartum [6].

The diagnosis of infectious sacroiliitis during pregnancy requires a degree of clinical suspicion and should be confirmed by imaging diagnostic methods. Plain radiography may give normal images in early disease. There may be blurring of joint margins, a widened joint space, or periarticular erosion [7]. Radioisotopic bone scans have high specificity and sensibility for localizing bone inflammation but should not be used during pregnancy. MRI is probably the imaging diagnosis method of choice in pregnancy to detect sacroiliitis. It provides a detailed evaluation of the joint and surrounding soft tissue without exposing the fetus to ionizing radiation [6]. We used MRI for imaging diagnosis method too. It revealed joint space widening and effusion of the right SIJ indicating acute right-sided sacroiliitis and also edema of the right psoas muscle. An ultrasound guided aspiration of the fluid was planned, but the patient could not be positioned due to the enlarged uterus.* Staphylococcus aureus* is the most common cause of infectious sacroiliitis. As we could not sample the liquid, we could not find the agent of infection in our case. Other conditions such as brucellosis or tuberculosis may produce sacroiliitis [8]. However, in both entities, clinical course is chronic. Embolic septic events in the setting of bacterial endocarditis may also be responsible for infectious sacroiliitis [9]. All of these conditions were excluded in our patient.

The treatment for pregnancy-related bacterial sacroiliitis is similar to that for non-pregnancy-related cases. Most authors recommend 4–6 weeks of parenteral antibiotic therapy [7]. We also used antibiotic therapy in our case.

There is no consensus on the appropriate way for delivery of patients with active pyogenic sacroiliitis [6]. Vaginal delivery could have been attempted in our patient. Epidural analgesia was considered to be contraindicated because of the risk of a disseminated infection to the spinal cord and meninges. Local or general anaesthesia might be other alternatives to relieve pain. As the patient was suffering severely from pain, the decision to perform a caesarean section was made on the basis of avoiding pain and joint distraction during delivery.

RETRACTED

In conclusion, sacroiliitis although uncommon should be considered in pregnant patients who present with acute severe localized pain and fever, even when no predisposing factors are detected. Delay in diagnosis and lack of therapy may result in severe complications. Pyogenic sacroiliitis complications include not only joint and bone destruction, but also maternal and neonatal septicaemia. Prompt diagnosis and treatment may avoid life-threatening complications for the mother and fetus.

## Figures and Tables

**Figure 1:** MRI images of right sacroiliac junction and sacroiliitis are shown by the arrow. Edema of right psoas muscle is shown by asterisk.

**Figure 2:** CT image of right sacroiliac junction after treatment.

## References

[1] Mens J. M. A., Vleeming A., Snijders C. J., Koes B. W., Stam H. J. (2001). Reliability and validity of the active straight leg raise test in posterior pelvic pain since pregnancy. *Spine*.

[2] Damen L., Buyruk H. M., Güler-Uysal F., Lotgering F. K., Snijders C. J., Stam H. J. (2001). Pelvic pain during pregnancy is associated with asymmetric laxity of the sacroiliac joints. *Acta Obstetricia et Gynecologica Scandinavica*.

[3] Vleeming A., Albert H. B., Östgaard H. C., Sturesson B., Stuge B. (2008). European guidelines for the diagnosis and treatment of pelvic girdle pain. *European Spine Journal*.

[4] Ostgaard H. C., Zetherstrom G., Roos-Hansson E., Svanberg B. (1994). Reduction of back and posterior pelvic pain in pregnancy. *Spine*.

[5] Egerman R. S., Mabie W. C., Eifrid M., Whitnack E., Sibai B. M. (1995). Sacroiliitis associated with pyelonephritis in pregnancy. *Obstetrics & Gynecology*.

[6] Jedwab M., Ovadia S., Dan M. (1999). Pyogenic sacroiliitis in pregnancy. *International Journal of Gynecology & Obstetrics*.

[7] Linnet K. M., Gammelgaard L., Johansen M., Krarup N., Rasmussen K. L. (1996). Bilateral pyogenic sacroiliitis following uncomplicated pregnancy and labor. *Acta Obstetricia et Gynecologica Scandinavica*.

[8] González-Gay M. A., García-Porrúa C., Ibañez D., García-País M. J. (1999). Osteoarticular complications of brucellosis in an atlantic area of Spain. *Journal of Rheumatology*.

[9] González-Juanatey C., González-Gay M. A., Llorca J. (2001). Rheumatic manifestations of infective endocarditis in non-addicts: a 12-year study. *Medicine*.

